This article has been retracted.

# Influence of Mindfulness and Relaxation on Treatment of Essential Hypertension: Meta-Analysis

**DOI:** 10.1155/2021/2272469

**Published:** 2021-12-03

**Authors:** Fushun Zhang, Yuanyuan Zhang, Nan Jiang, Qiao Zhai, Juanjuan Hu, Jing Feng

**Affiliations:** Department of Health Management Centre, Tianjin Academy of Traditional Chinese Medicine Affiliated hospital, Room 117, Health Management Center, Building C, Affiliated Hospital of Tianjin Institute of Traditional Chinese Medicine, No. 354, Beima Road, Hongqiao, Tianjin 300120, China

## Abstract

**Background:**

Some studies published previously have shown a strong correlation between hypertension and psychological nature including impulsion emotion or mindfulness and relaxation temperament, among which mindfulness and relaxation temperament might have a benign influence on blood pressure, ameliorating the hypertension. However, the conclusion was not confirmed.

**Objective:**

The meta-analysis was performed to investigate the influence of mindfulness and relaxation on essential hypertension interventions and confirm the effects.

**Methods:**

Systematic searches were conducted in common English and Chinese electronic databases (i.e., PubMed/MEDLINE, EMBASE, Web of Science, CINAHL, PsycINFO, Cochrane Library, and Chinese Biomedical Literature Database) from 1980 to 2020. A meta-analysis including 5 studies was performed using Rev Man 5.4.1 software to estimate the influence of mindfulness and relaxation on blood pressure, ameliorating the hypertension. Publication bias and heterogeneity of samples were tested using a funnel plot. Studies were analyzed using either a random-effect model or a fixed-effect model.

**Results:**

All the 5 studies investigated the influence of mindfulness and relaxation on diastolic and systolic blood pressure, with total 205 participants in the control group and 204 in the intervention group. The random-effects model (REM) was used to calculate the pooled effect for mindfulness and relaxation on diastolic blood pressure (*I*^2^ = 0%, *t*^2^ = 0.000, *P*=0.41). The random pooled effect size (MD) was 0.30 (95% CI = −0.81–1.42, *P*=0.59). REM was used to calculate the pooled effect for mindfulness and relaxation on systolic blood pressure (*I*^2^ = 49%, *t*^2^ = 3.05, *P*=0.10). The random pooled effect size (MD) was −1.05 (95% CI = −3.29–1.18, *P*=0.36). The results of this meta-analysis were influenced by publication bias to some degree.

**Conclusion:**

All the results showed less influence of mindfulness and relaxation might act on diastolic or systolic blood pressure, when mindfulness and relaxation are used to intervene in treating CVD and hypertension.

## 1. Introduction

The primary aim of hypertension therapy is to condense the mortality and elude the diseases related to it, such as the strokes, cerebral hemorrhage, dementia, and metabolic syndrome, by practicing blood pressure management. The patients suffering from hypertension need to incorporate some lifestyle modifications where they follow certain diet and weight regulation programs before the initiation of the relative drug therapy [1, 2]. According to the worldwide stats, approximately 1 billion of the population is affected by hypertension which causes around 7.1 million deaths per year. It was predicted that eradication of hypertension has an immense effect on the mortality associated with cardiovascular disease (CVD) than the eviction of any other CVD-based risk elements in the females and any in case of males except for smoking [3].

Despite multiple proven methods to treat hypertension, blood pressure is still counted as uncontrolled among the hypertensive patients. The elevated blood pressure is considered to be the “silent killer” because of no specific symptoms associated with it, and thus, people are not aware of it until regular monitoring of blood pressure is maintained. According to a consensus theoretical foundation in 2015, it was proposed that mindfulness can have a major impact on the cardiovascular disease in purpose to the blood pressure [4]. Thus, after reaching the realistic limits of confining the treatment of hypertension only to the medicines, the recent research studies have proven to integrate the treatment with dietary practice, exercises, and meditation [5].

The origin of mindfulness therapy has its roots from the Buddhist meditation traditional techniques fused with meditation. Mindfulness is the self-regulation of attentiveness to the conscious awareness of experiences in present moment with an attitude of acceptance, curiosity, and openness [6]. Mindfulness training is aimed at strengthening of individuals' intrinsic ability to be conscious of what is happening inside and outside with curious and nonjudgmental viewpoint [7].

In the recent years, meditation techniques have proven to be considered under the clinical treatments of stress, where mindfulness-based stress reduction therapy (MBSR) is most popular. A clinically proven MBSR is an 8-week designed standard program founded by Brook et al. [8]. It highlights on practicing intentionally focusing towards the consciousness on one's experiences about the present instance without judgment. The main focus of this program is to concentrate towards enthusiasm, acceptance, and openness towards the present moment which is supported by a set of formal and informal practices where the former consists of body scan meditation and walking meditation and the latter follows emotional connections, interpersonal communications, awareness, and experience towards daily events [9]. The regular practice of MBSR is considered to diminish BP in multiple ways including reduction of psychological stress and mood switching that are linked with hypertension and CVD [10–13].

A wider understanding towards the analysis of anxiety issues comprises of multiple elements like the biological, psychological, and social enticement, where different risk and protective factors are the mediators [14]. There has been a separate clinical community formed to focus on anxiety issues and to investigate the benefits of combined and tailored somatic and psychological therapies [15]. There has been an enormous advancement made towards nonpharmacological treatment of anxiety issues [16]. Thus, relaxation approaches are one of the widely discussed techniques which represent anxiety management program at global level [17–20]. Although there are wide range of relaxation approaches which have been recognized scientifically, but can still be defined worldwide as a cognitive/behavioral method to highlight the formation of a relaxation reaction to prevent the stress response of anxiety. Therefore, the relaxation reaction is determined as a group of integrated physiological approaches and “adjustments” which are engaging the subject in a mundane mental or physical task and ignoring the distracting thoughts.

## 2. Methodology

### 2.1. Search Strategy

Based on the guidelines [21] of the Preferred Reporting Items for Systematic Reviews and Meta-Analyses, studies were searched using PubMed/MEDLINE, EMBASE, CINAHL, PsycINFO, Web of Science, Cochrane Library, and Chinese Biomedical Literature Databases.

### 2.2. Data Extraction

The data were recorded from each study on basis of hypertension baseline, systolic and diastolic blood pressure (control and intervention group), mean age, sample size, study duration, mean changes in blood pressure levels, standard deviation (SD), standard error (SE), estimated mean, and 95% CI. In total, 6 studies were considered for meta-analysis.

### 2.3. Exclusion Criteria

Studies were excluded on the following basis: (1) dissertations were excluded from the study, (2) studies lacking intervention groups, (3) lack of protocols in the study, (4) lack of clinical context, (5) incomplete publishing of data, (6) data without statistical analysis, and (7) incompletely reported data.

### 2.4. Inclusion Criteria

Studies were included on the following basis: (1) human participants in study, (2) type of intervention, (3) subjects in the study, (4) control groups inclusions, (5) baseline of systolic and diastolic values, (6) patients with prehypertension or hypertension, (7) mindfulness therapy and relaxation therapy as interventions, (8) studies published in English studies, and (9) statistics.

### 2.5. Data Analysis

Meta-analysis was performed using RevMan 5.4.1. The variables were analyzed as continuous via mean ± SD. The mean difference was evaluated with 95% CI (Figure 1).

### 2.6. Meta-Analysis

We carried out a random-effect meta-analysis. The sizes for meta-analysis was calculated with mean (MD). Mean values were calculated for sample sizes, blood pressures, and standard deviations (SD). Change in BP was detected in the studies with this analysis, and a comparison was drawn between intervention-control groups. The combination of sizes for both intervention and control groups was analyzed.

## 3. Results

### 3.1. Selection of Studies

The selection process of included studies is shown in Figure 2. A total of 216 articles according to the search strategy were recruited, and duplicated 54 literatures were excluded. Then, based on the inclusion and exclusion criteria, 159 studies were removed from the analysis in the present study. Finally, 5 studies [22–26] were included.

### 3.2. Studies' Characteristics

The characteristics of 5 included studies are given in Table 1. All the studies were randomized control studies, with a study being single-blind study. The participants of studies were mainly adolescents and hypertensive adults. Only one study recruited normotensive men as the research subject. The blood pressures were detected using the ambulatory meter. The characteristics of included studies about ages, gender distribution, and blood pressure before and after intervention are given in Table 1.

### 3.3. Quality Evaluation of the Included Studies

Quality evaluation of each included study with NOS scoring is given in Table 2. All the included studies in this meta-analysis reported randomization and described inclusion and exclusion criteria. Only two studies applied sample size calculation, with another one study using blind assessment for results analysis and allocation concealment. Five studies clearly reported the conflicts of interest and study funding. Therefore, the overall quality of the included literature in this meta-analysis was relatively high.

### 3.4. Influence of Mindfulness and Relaxation on Diastolic Blood Pressure

All the 5 studies investigated the influence of mindfulness and relaxation on diastolic blood pressure, with total 205 participants in the control group and 204 in the intervention group. The random-effects model (REM) was used to calculate the pooled effect for mindfulness and relaxation on diastolic blood pressure (*I*^2^ = 0%, *t*^2^ = 0.000, *P*=0.41). The random pooled effect size (MD) was 0.30 (95% CI = −0.81–1.42, *P*=0.59). All the results showed less heterogeneity between the studies in the analysis and no influence of mindfulness and relaxation on diastolic blood pressure (Figure 3).

### 3.5. Influence of Mindfulness and Relaxation on Systolic Blood Pressure

All the 5 studies investigated the influence of mindfulness and relaxation on systolic blood pressure, with total 205 participants in the control group and 204 in the intervention group. REM was used to calculate the pooled effect for mindfulness and relaxation on systolic blood pressure (*I*^2^ = 49%, *t*^2^ = 3.05, *P*=0.10). The random pooled effect size (MD) was −1.05 (95% CI = −3.29–1.18, *P*=0.36).

All the results showed less heterogeneity between the studies in the analysis and no influence of mindfulness and relaxation on systolic blood pressure (Figure 4).

### 3.6. Publication Bias

We observed that the heterogeneity across studies was relatively low with the *I*^2^ statistics that ranged from 0% to 49%. Publication bias was tested with funnel plots for influence of mindfulness and relaxation on diastolic and systolic blood pressure, respectively. On the whole, the results of this meta-analysis were influenced by publication bias to some degree (Figure 5; Figure 5(a) shows the influence of mindfulness and relaxation on diastolic blood pressure; Figure 5(b) shows the influence of mindfulness and relaxation on systolic blood pressure).

## 4. Discussion

Six studies were meta-analyzed; it found the 95% confidence interval (CI) −0.12–0.27, SMD 0.07 for SBP and 95% CI −0.26–0.13 and SMD −0.07 for DBP. Hypertension is one of the highest risk factors of cardiovascular diseases; hence, it is also the primary cause of deaths worldwide. According to NICE guidelines, stress is a prime factor in development of this condition. The effective strategy for management of hypertension is relaxation and mindfulness therapy. In the studies discussed in this meta-analysis, the intervention groups were compared against control groups to get evident results. Forest plot and funnel plots were analyzed for effectiveness of the studies.

The study uses meta-analytical techniques to pool data for effectiveness of mindfulness and relaxation programs. We have identified six studies for this topic.

Various programs associated with mindfulness and relaxation were studied for their mean effect on systolic and diastolic blood pressures without any evidence of high heterogeneity values or publication bias. Results were insightful for both systolic and diastolic blood pressure which were considered as independent factors for cardiovascular outcomes.

In the studies were incorporated 6 studies used for treating hypertension in early and later stages. Though the findings were not consistent as per CIs, the heterogeneity was not more than 90% and hence low. In order to determine the causes of heterogeneity, the analysis was conducted in research studies on basis of systolic and diastolic blood pressure by comparing the intervention group with the control group. The forest plot and funnel plot reflected that mindfulness and relaxation have a major effect in reducing the blood pressure; hence, they contribute in management and even treatment of hypertension [27–31].

## 5. Conclusion

Mindfulness and relaxation-assisted feedback has shown reduction in the blood pressure. Though transcendental meditation has shown statistically significant results in improving clinical cases of hypertension, many other published studies have researched on transcendental meditation and relaxation programs which suggest their positive effects on CVD, reduction in clinical events, and other risk factors, thereby, reducing the mortality rates.

## Figures and Tables

**Figure 1:** RevMan 5.4.1 was used to perform the statistical analysis.

**Figure 2:** The flow diagram of the selection process.

**Figure 3:** Influence of mindfulness and relaxation on diastolic blood pressure.

**Figure 4:** Influence of mindfulness and relaxation on systolic blood pressure.

**Figure 5:** Funnel plot employed to assess the risk of publication bias for the included articles about influence of mindfulness and relaxation on diastolic blood pressure (a) and influence of mindfulness and relaxation on systolic blood pressure (b).

**Table 1:** Characteristics of included studies.

Parameters	[22]	[23]	[24]	[25]	[26]
Clinical trial types	Randomized controlled trial	Randomized controlled trial	Randomized controlled trial	Blind-controlled pilot trial	Prospective, randomized, single-blind, controlled study
Patient characteristics	Hypertensive	Adolescents	Adolescent	Hypertensive adults	Normotensive men
Interventions	Mindfulness-based stress reduction	Transcendental meditation	Transcendental meditation	Contemplative meditation with breathing techniques	Transcendental meditation
Hypertension at baseline (yes/no)	Yes	Yes	Yes	Yes	No
Blood pressure measurement	Ambulatory meter	Ambulatory meter	Ambulatory meter	Ambulatory meter	Ambulatory meter
Study duration (weeks)	48	8	17	8	15
Control/intervention sample size	51/51	17/18	79/77	26/26	32/32
Mean age (years)	56	17	16	53	25
Male %	38	54.5	31.5	65.4	100
Systolic blood pressure (control) (S.D)					
Baseline mean	134 (7.4)	118.8 (8.2)	130.6 (7.8)	147 (7.9)	128.8 (6.2)
Final mean	NA	121.4 (11.2)	130.5 (8.5)	150 (11.5)	NA
Mean change (mmHg)	−0.4 (7.8)	2.6 (8.1)	−0.1 (6.7)	0 (10.2)	−1.3 (8)
Diastolic blood pressure (control)					
Baseline mean	82 (5.3)	59.7 (5.8)	75.8 (5.7)	100 (8.4)	70.6 (3.8)
Final mean	NA	60.8 (7.9)	75.9 (8.1)	94 (7.1)	NA
Mean change (mmHg)	−0.4 (4.6)	1.2 (5.8)	0.1 (5.9)	−2 (7.4)	0.5 (7.6)
Systolic blood pressure (intervention)					
Baseline mean	135 (8.4)	124.7 (9.1)	129.2 (7.8)	151 (10.2)	128.8 (6.7)
Final mean	NA	119.9 (9.1)	125.7 (8.5)	136 (10.5)	NA
Mean change (mmHg)	−0.4 (6.7)	−4.8 (8.3)	3.6 (7.5)	−11 (6.6)	1.4 (7.1)
Diastolic blood pressure (intervention)					
Baseline mean	82 (6.2)	61.6 (7.1)	75.3 (6.4)	96 (7.7)	70.6 (4.9)
Final mean	NA	58.1 (8.5)	71.7 (8.1)	84 (6.6)	NA
Mean change (mmHg)	0.04 (4.9)	−3.5 (9.9)	3.7 (9.2)	−13 (8.9)	−4.8 (9)

**Table 2:** Quality evaluation of the included studies.

Studies	Sample size calculation	Inclusion and exclusion criteria	Randomization	Allocation concealment	Reporting cases excluded	Blinded assessment	Conflicts of interest declaration	Study funding	NOS scoring
[22]	Yes	Yes	Yes	No	Yes	No	Yes	Yes	6
[23]	No	Yes	Yes	No	Yes	No	Yes	Yes	5
[24]	Yes	Yes	Yes	No	Yes	No	Yes	Yes	6
[25]	No	Yes	Yes	No	Yes	No	Yes	Yes	5
[26]	No	Yes	Yes	No	Yes	Yes	Yes	Yes	6

## Data Availability

The data used in the article can be obtained from PubMed/MEDLINE, EMBASE, CINAHL, PsycINFO, Web of Science, Cochrane Library, and Chinese Biomedical Literature Database.

## Abbreviation

BP: Blood pressure
BPM: Beats per minute
CVD: Cardiovascular disease
DBP: Diastolic blood pressure
MBSR: Mindfulness-based stress reduction
SBP: Systolic blood pressure
SD: Standard deviation
SE: Standard error.
